# Development of a Bile Acid-Related Gene Signature for Predicting Survival in Patients with Hepatocellular Carcinoma

**DOI:** 10.1155/2022/9076175

**Published:** 2022-05-10

**Authors:** Gang Wang, Jun Guan, Qin Yang, Fengtian Wu, Junwei Shao, Qihui Zhou, Zixuan Guo, Yanli Ren, Haihong Zhu, Zhi Chen

**Affiliations:** Key Laboratory for Diagnosis and Treatment of Infectious Diseases, National Clinical Research Center for Infectious Diseases, National Medical Center for Infectious Diseases, Collaborative Innovation Center for Diagnosis and Treatment of Infectious Diseases, The First Affiliated Hospital, Zhejiang University School of Medicine, Hangzhou, China

## Abstract

**Background:**

Hepatocellular carcinoma (HCC) is one of the most common diseases that threaten millions of lives annually. Evidence supports that bile acid (BA) affects HCC through inflammation, DNA damage, or other mechanisms.

**Methods:**

A total of 127 BA-associated genes were analyzed in HCC tumor and nontumor samples using The Cancer Genome Atlas data. Genes correlated to the prognosis of patients with HCC were identified using univariate and multivariate Cox regression analyses. Furthermore, a prediction model with identified genes was constructed to evaluate the risk of patients with HCC for prognosis.

**Results:**

Out of 26 genes with differential expressions between the HCC and nontumor samples, 19 and 7 genes showed upregulated and downregulated expressions, respectively. Three genes, NPC1, ABCC1, and SLC51B, were extrapolated to construct a prediction model for the prognosis of patients with HCC.

**Conclusion:**

The three-gene prediction model was more reliable than the pathological staging characters of the tumor for the prognosis and survival of patients with HCC. In addition, the upregulated genes facilitating the transport of BAs are associated with poor prognosis of patients with HCC, and genes of de novo synthesis of BAs benefit patients with HCC.

## 1. Introduction

Liver cancer is one of the most common cancers worldwide and the third highest cause of cancer mortality, with 0.84 million new cases and 0.78 million deaths annually [1]. China has vast cases of hepatitis B virus (HBV) infections, resulting in a high incidence of liver cancer and one of the leading causes of cancer deaths in China [2]. Increased incidence rates of liver cancer, among other cancers, have been reported [3]. Seventy percent of the whole blood supply in the liver is circulated from the portal vein, where the blood is transported from the intestine, containing nutrients, metabolites, products of gut bacteria, and bile acid (BA) [4].

In the past decades, more investigations are emerging on the correlations between gut microbiota and hepatocellular carcinoma (HCC) [5, 6]. The gut microbiota produces numerous metabolites in the human body, including lipopolysaccharides (LPS), short-chain fatty acids, and BAs, which could promote haptic inflammation, resulting in liver diseases such as liver fibrosis, liver cirrhosis, and HCC [5]. Among the metabolites, BAs are vital components of enterohepatic cycling, a cycle between the enterointestine and the liver that maintains BAs for the homeostasis of cholesterol and human nutrient uptake [7–10]. BAs are a group of heterogeneous cholanic acids with steroid nuclei, consisting of cholic acid (CA), chenodeoxycholic acid (CDCA), deoxycholic acid (DCA), lithocholic acid (LCA), and ursodeoxycholic acid (UDCA). CA, CDCA, DCA, and LCA are free BAs conjugated by glycine (G) or taurine (T) to formulate (G/T)-(CA/CDCA/DCA/LCA)-conjugated BAs, which are the main components in human BAs [11]. BAs are primarily synthesized from cholesterol through multiple modified enzymatic steps involving 17 enzymes, including rate-limiting enzymes cholesterol 7*α*-hydroxylase (CYP7A1), sterol 27A-hydroxylase (CYP27A1), and oxysterol and steroid 7*α*-hydroxylase (CYP7B1), as well as other enzymes in hepatocytes (reviewed in [11]). BAs form the majority of solid components in gallbladder bile, such as sodium (Na^+^) and potassium (K^+^) salts of the BAs [11, 12].

In humans, bile, including BAs and other constituents, is stored in the gallbladder and released after a meal into the intestinal lumen as emulsifiers to solubilize fats and fat-soluble vitamins and facilitate nutrient uptake [8, 12]. In the human intestine, 95% of BAs are absorbed in the intestinal blood and circulated in the liver through the portal vein [13]. In the liver, several transporters are involved in the cross-membrane transport of BAs within the gut-liver-gallbladder circle. In the gut, the ileum uptakes most BAs (~95%) via the apical sodium-dependent BA transporter, after which the BAs are exported in the portal vein via organic solute transporter *α* and *β* heterodimers (OST*α*/OST*β*) [14]. In the liver, hepatocytes uptake BAs from the venous blood via Na^+^-dependent Na^+^ taurocholate cotransporting polypeptide (NTCP/SLC10A1) and Na^+^-independent organic anion transporting polypeptide (OATP) family members (OATP-A/SLC21A3, OATP-C/SLC21A9, and OATP-8/SLC21A8 in humans) [15]. The BA efflux in hepatocytes involves the multidrug resistance protein (MRP) subfamily, such as MRP-1, MRP-2, MRP-3, and MRP-6 [15]. In addition, bile canalicular excretion of BAs requires two types of transporters that pump BAs out, such as bile salt export pump (BSEP) (ABCB11) and ATP-binding cassette (ABC) superfamily members, including ABCA (1, 2, and 3), ABCG (2, 5, and 8), and MRP2 (ABCC2) [15].

The BA synthesis or recycling process disorder could result in diseases such as gallstones, obesity, liver diseases, and other metabolic syndromes [16–18]. Furthermore, BAs initiate signaling pathways and induce cellular injuries in many cancers, including liver cancer [19–22]. Several reports suggest that BAs have critical roles in cell proliferation, inflammation, cell invasion, cellular metabolism, and other cellular behaviors [20, 21, 23, 24]. Here, we explore the genes involved in metabolic pathways and transportation systems of BAs in liver cells to find significant markers for the prognosis and survival of patients with HCC.

## 2. Materials and Methods

### 2.1. Genes Involved in the Transport and Metabolism of BAs

The list of BA metabolic genes was obtained from Gene Set Enrichment Analysis (GSEA) (http://software.broadinstitute.org/gsea/msigdb, file name: Bile acids metabolism gene set, 112 genes) [25]. Fifteen genes involved in the transporters for hepatocyte influx and BA outflux, such as ABCB11, ABCC1, ABCC2, ABCC3, ABCC6, ABCG2, ABCG5, SLC10A1, SLC10A2, SLC51A, SLC51B, SLCO1B3, SLCO2B1, and BA syntheses, such as ACOT8 and BAAT, were added to the list [15]. Hence, 127 BA-associated genes were included in the present study (Table S1).

### 2.2. Data Acquisition

The data of patients with HCC was downloaded from The Cancer Genome Atlas (TCGA) (https://portal.gdc.cancer.gov/) and focused on TCGA-liver hepatocellular carcinoma data. In total, 424 sample sequencing and 377 clinical data files of patients with HCC were downloaded. All patients with HCC had completed clinical characteristics and follow-up data (≥1 month). Among the sequencing samples, 50 nontumor samples and 374 HCC samples were used to analyze the differential expressions of BA-associated genes. The follow-up time was used to evaluate the effects of BA-associated genes on the survival of patients with HCC. *P* value < 0.05 and fold change > ∣2∣ were considered significant.

### 2.3. Data Processing

The Perl software (version 5.28) and R software (version 4.0) were employed for data processing. The Perl software (version 5.28) was used to combine the clinical and gene expression data based on patient IDs as well as merge the splicing files of individual samples or patients.

The R software (version 4.0) with the “limma” package was used to identify the BA-associated genes with differential expressions between the tumor and nontumor groups. For the probability of type I error, an adjusted *P* value of <0.05 and the fold change of >|2| were significant for differential gene expression [26, 27]. The heatmap, volcano, and boxplot graphs were constructed using packages “pheatmap,” “limma,” and “ggpubr” to illustrate the gene levels.

Gene enrichment and annotation with Gene Ontology (GO) terms and Kyoto Encyclopedia of Genes and Genomes (KEGG) pathways were performed using the R software with “clusterProfiler,” “http://org.Hs.eg.db/,” “enrichplot,” “ggplot2,” or “GOplot” packages. Adjusted *P* value of <0.05 was significant for annotation and enrichment of GO terms and KEGG pathways [28, 29].

### 2.4. Construction of a Prediction Model for the Prognosis of Patients with HCC

The survival analysis of the identified genes was analyzed using packages “survival” and “survminer” in R. The receiver operating characteristic (ROC) curve to predict the prognostic value was analyzed using the “survivalROC” package in R.

Univariate Cox regression analysis was used to explore the correlation between gene expression and patient survival (*P* < 0.05). Multivariate Cox regression analysis was used to identify the BA-associated genes that were candidate genes to construct the prediction model. The coefficients of the selected genes were used to construct the model. The risk score of every patient is equal to coefficient1 × expression value of gene1 + coefficient2 × expression value of gene2 + coefficient(*n*) × expression value of gene(*n*) (Table S2). Based on the median value of the risk score, the patients were divided into the high-risk and low-risk groups. Two packages in R, “survival” and “survminer,” were employed to construct the survival curve of the two groups. The timeline of the ROC curve was from 0 to 10 years. The ROC curve with high- and low-risk groups was constructed under a timeline of multiple years using clinical characteristics, including age, gender, stage, grade, and TNM, and the risk score model.

### 2.5. Correlation Analysis of Clinical Characteristics and Model Genes

According to gender (male and female), stage (I, II, III, and IV), grade (1, 2, 3, and 4), and TNM (tumors (T), nodes (N), and metastases (M)), patients with HCC were divided into two groups. The expression values of the three genes in the prediction model and risk scores of patients in each group were statistically analyzed for significant differences. *P* value < 0.05 was considered significant.

### 2.6. Immunohistochemistry

Anti-SLC51B antibody (Cat. ab121285) and Niemann Pick C1 antibody (Cat. ab134113) were purchased from Abcam (Cambridge, USA), and MRP1/ABCC1 antibody (Cat. 72202) was purchased from Cell Signaling Technology Inc. The liver tumor tissue array was purchased from Superchip, Inc. (Shanghai, China). The immunohistochemistry procedures were performed as described in previous work [30].

### 2.7. Statistical Analyses

All statistical analyses were performed using R software with various packages, with *P* value < 0.05 or 0.01 considered significant. KEGG and GO analysis used the adjusted *P* value < 0.05 as significant. Further, the Wilcoxon test was used to identify differentially expressed BA-associated genes.

## 3. Results

### 3.1. Identification of 26 BA-Associated Genes with Significant Differential Expressions between the Tumor and Nontumor Samples of Patients with HCC

To explore differential gene expressions in the metabolism and transport of BAs in patients with HCC, 112 genes from the GSEA website and 15 genes associated with the metabolism and transport of BAs in the liver were downloaded, resulting in 127 genes (Table S1). The expressions of 127 genes in tumor and nontumor samples and 26 genes, including ABCA2, ABCA3, ABCA4, ABCC1, ABCD1, ACSL1, AKR1D1, ALDH8A1, BBOX1, CYP39A1, CYP7A1, DIO2, EFHC1, FADS1, FADS2, GNPAT, KLF1, LIPE, NPC1, PEX6, PFKM, SLC27A5, SLC29A1, SLC35B2, SLC51B, and SLCO1B3, were identified under the criteria of fold change > ∣2∣ and adjusted *P* value < 0.05 (false discovery rate (FDR) < 0.05) (Figure 1(a)) [27]. Among the identified genes, 19 genes (ABCA2, ABCA3, ABCA4, ABCC1, ABCD1, CYP7A1, DIO2, EFHC1, FADS1, FADS2, GNPAT, KLF1, LIPE, NPC1, PEX6, PFKM, SLC29A1, SLC35B2, and SLC51B) and 7 genes (ACSL1, AKR1D1, ALDH8A1, BBOX1, CYP39A1, SLC27A5, and SLCO1B3) were upregulated in the tumor and nontumor samples, respectively (*P* < 0.05) (Figures 1(b) and 1(c)). The results suggested that most genes with differential expressions were transporter proteins, such as solute carrier (SLC) and ATP-binding cassette (ABC) family proteins, which carry BAs or other metabolic mediates shuttling in the liver.

### 3.2. Annotation and Enrichment of Identified Genes Using GO and KEGG Analyses

The functions and pathways involved in the 26 identified genes were further explored using GO and KEGG functional enrichment analyses (adjusted *P* value < 0.05). These genes were associated with primary BA biosynthesis, ABC transporters, the PPAR signaling pathway, and monocarboxylic acid synthesis. The details are shown in Figure 2 and Fig. S1. The enrichment analysis and annotation showed that the genes with upregulated differential expressions in patients with HCC were associated with ABC transporters, cholesterol metabolism and biosynthesis of fatty acids (KEGG), and lipid transport and localization (GO). The genes with downregulated differential expressions in patients with HCC were associated with the BA metabolism process (GO) and primary BA biosynthesis (KEGG) (Figure 2 and Fig. S2). In addition, a few genes were associated with the PPAR signaling pathway, peroxisome, and metabolism of sterol. These results indicate that reduced BA synthesis and increased BA and lipid transporters, including fatty acids, have vital roles in HCC.

### 3.3. Identification of Survival-Related Genes Associated with BA Metabolism

To examine whether the identified genes had effects on survival time, a univariate Cox regression analysis was performed using the “survival” package in R (cutoff value: *P* < 0.05). A total of 376 patients with HCC with follow-up time were included in the study. Consequently, 12 genes were identified, 4 of which (SLC27A5, CYP7A1, AKR1D1, and ALDH8A1) benefitted the patients while the remaining 8 (EFHC1, ABCC1, NPC1, ABCD1, SLC35B2, ABCA4, ABCA3, and SLC51B) increased the risk of poor prognosis (Figure 3). Furthermore, a multivariate Cox regression analysis was performed for all 25 genes. Three genes, NPC1, ABCC1, and SLC51B, showed significant relationships with the survival time of patients with HCC (Figure 4(a) and Table 1). These results suggest that high expressions of NPC1, ABCC1, and SLC51B may increase the risk of poor prognosis, resulting in a negative correlation with the survival of these patients (hazard ratios of 1.48, 1.30, and 1.16, respectively). In addition, these three genes were detected on HCC tissue immunohistochemistry and showed higher expression levels compared to the control tissues (Fig. S3).

### 3.4. Construction of a Prediction Model for the Prognosis of HCC in Patients

Based on the multivariate Cox regression analysis, the three identified genes were employed to construct a prediction model for the risk of poor prognosis of HCC in patients. The risk score for each patient was calculated as follows: risk score = (0.396 × value of NPC1 expression) + (0.262 × value of ABCC1 expression) + (0.155 × value of SLC51B expression). Accordingly, all patients with HCC had risk score values (Table 1). Following the median values of the ranked risk scores, the patients were divided into the high-risk and low-risk groups (Figure 4(b)). The time-dependent distribution of the status of these patients showed an increase in the number of deceased patients with time (Figure 4(c)). Accordingly, the Kaplan–Meier survival curve showed that the patients with high risk scores had higher mortality rates than those with low risk scores (log-rank *P* = 4.47 × 10^−6^). The low-risk and high-risk groups had different 3-year (74.8% and 48.2%, respectively, *P* < 0.01) and 5-year survival rates (55.7% and 38.5%, respectively, *P* < 0.01) (Figure 4(d)).

### 3.5. Three-Gene Risk Model Is More Reliable for Prediction of Prognosis

The efficiency of the prediction model was examined. The risk scores of the model and clinical or pathological characteristics of patients with HCC were included in the univariate and multivariate Cox regression analyses. The clinical data contains three cancer staging types: cancer grade, cancer stage, and TNM staging. In the present study, most cases of HCC were N0 and M0, according to the TNM staging system. Hence, the pathology grouping characteristics included stages, grades, and T without corresponding to N (whether patients had invading local lymph nodes) and M (whether patients had metastases). Univariate analysis demonstrated that stages, T, and risk scores were significantly correlated with the prognosis of HCC in patients (all *P* < 0.01) (Figure 5(a)). However, multivariate analysis showed that only risk scores were significantly associated with the prognosis of such patients (*P* < 0.001, hazard ratio = 1.568, and 95% CI: 1.256–1.956) (Figure 5(b)). Furthermore, a ROC curve and the area under the curve (AUC) were performed to evaluate the probability of the prediction model. The ROC curve confirmed that the risk score prediction system (AUC = 0.710) was more reliable in predicting the prognosis of HCC in patients than the cancer staging system (Figure 5(c)).

### 3.6. Analysis of the Correlation between Model Genes and Clinical Characteristics

NPC1, ABCC1, and SLC51B genes were identified in the prediction model. There are five clinical characteristics such as age, gender, and three cancer staging systems, including stage (0, I, II, III, and IV), grade (1, 2, 3, and 4), and TNM [31]. Each clinical characteristic was divided into two groups according to gender (male and female), age (<65 y and ≥65 y), stage (stage I–II and stage III–IV), grade (grade 1–2 and grade 3–4), and TNM (T1–2 and T3–4) (Figure 6). No significant differential expressions were observed for age and gender in the three genes (*P* > 0.05). Cancer staging systems in NPC1 showed high differential expressions for stage (stages III–IV, *P* < 0.001), grade (grades 3–4, *P* < 0.001), and TNM (T3–4, *P* < 0.001) in patients with HCC (Figures 6(a)–6(c)). Similarly, cancer staging systems in ABCC1 showed high differential expressions for the grade, stage, and T (*P* = 0.014, *P* = 0.008, and *P* = 0.016, respectively) in patients with HCC (Figures 6(d)–6(f)). In addition, no differential expressions were observed in SLC51B among different stages of HCC. Furthermore, the risk scores of the patients in different cancer staging groups were compared, which showed that the risk scores increased with the higher pathological stagings of HCC. Moreover, worse severity of HCC staging was associated with higher risk scores in different groups of the stage, grade, and T (*P* = 0.026, *P* < 0.001, and *P* = 0.027, respectively) (Figures 6(g)–6(i)). The data showed that NPC1 and ABCC1 increased expressions with the latter stages of HCC. The increasing risk score of the prediction model was associated with that of the stages of HCC.

## 4. Discussion

Although increasing reports suggest the involvement of enterohepatic circulation in the carcinogenesis of HCC, only a few studies have reported on the correlation between the genes involved in the transport and metabolism of BAs in the liver and HCC [32–34]. In the present study, 26 BA-associated genes with differential expressions were identified between the tumor and nontumor tissues collected from 127 genes (Figure 1). Eleven and three genes were identified using univariate and multivariate Cox regression analyses, respectively, which were significant for the prognosis of HCC in patients. These genes are involved in the metabolism and transport of BAs, cholesterol, and fatty acids (Figure 2). Subsequently, a prediction model for the survival of patients with HCC was constructed using NPC1, ABCC1, and SLC51B. The model value (risk score) was more reliable than the tissue pathological characteristics, such as tumor staging, TNM, and grading, in predicting the prognosis of HCC in patients (Figure 5).

Among the 26 differentially expressed genes, 19 genes showed high differential expressions, whereas 7 showed low differential expressions in HCC. Most downregulated genes were related to catalytic enzymes that participate in BA biosynthesis or upstream molecules, such as cholesterol and fatty acids. SLC27A5 aids in the formation of conjugated BAs (glycine-/taurine-BAs), AKR1D1 catalyzes a crucial step in the alternative pathway of BA synthesis, and CYP39A1 aids in the synthesis of cholesterol [8, 11, 35, 36]. Moreover, ACDL1 and BBOX1 aid in the synthesis and transport of lipids in liver cells, respectively [37, 38]. Most upregulated genes encode transporter proteins, including ABC family members, SLC family members, and NPC1. These transporters help transport BAs resorbed from portal vein blood into and out of liver cells [18]. In addition, BAs and their associated molecules require transporters to shuttle them into different compartments in cells. These transporters, including NTCP (SLC10A1), OATP1 (SLCO1A2), OATP2 (SLC21A6), OST*α* (SLC51A), OST*β* (SLC51B), MRP3 (ABCC3), MPR4 (ABCC4), MRP2 (ABCC2), BSEP, and MDR1A, are involved in lipid and cholesterol metabolism.

After examining the BA-associated genes and the prognosis of HCC in patients, 12 and 3 genes were identified using univariate and multivariate Cox regression analyses, respectively. Among the 12 genes, 4 showed negative correlations, and 8 showed positive correlations with the prognosis of HCC in patients. CYP7A1 and SLC27A5 were the most important genes controlling the classic and alternative ways of BA synthesis [10–12, 33]. In addition, AKR1D1 was a catalytic enzyme in BA synthesis [11]. ALDH8A1 is involved in the metabolism of tryptophan, which is linked to the metabolisms of fatty acid and cholesterol [39]. Evidence suggests that evaluating the de novo synthesis of BAs is beneficial to patients with HCC. Among the eight genes, ABCC1, ABCA3, ABCA4, SLC35B2, SLC51B, ABCD1, and NPC1 were transporter proteins, and EFHC1 was a calcium regulator protein [40]. The results indicated that continuous transportation of BAs in the enterohepatic cycle potentially deteriorated the condition of patients with HCC. NPC1, ABCC1, and SLC51B were determined using the multivariate Cox regression analysis to construct a prediction model for the prognosis of HCC in patients, and the risk scores of the patients were evaluated. These three genes were signatures for the prediction of the prognosis of HCC in patients.

BAs effectively facilitate the digestion and absorption of lipids, nutrients, lipid-soluble vitamins, and drugs. They also regulate the homeostasis of cholesterol and are recyclable during the digestive phase [11, 41]. The de novo synthesis of BAs is initiated by cholesterol and catalyzed by CYP7A1 or CYP27A1 (and CYP7B1) and other enzymes, resulting in the modification of the side chain and steroid nucleus and completing with CA and CDCA [11, 18, 41]. CA and CDCA conjugated to glycine and taurine form glycine-/taurine-cholic acid and glycine-/taurine-chenodeoxycholic acid [33]. The gut bacteria convert primary BAs to secondary BAs, such as DCA, UDCA, and LCA [14, 33]. In hepatic sinusoids, BAs are transported to hepatocytes using transporter proteins such as NTCP and OATP, sustaining the balance of the BA pool in the liver [18]. Simultaneously, the remaining part in the feces gets replenished by the newly synthesized BAs [33]. All BAs are discharged in the bile duct by transporters such as MRP2 and MDR1A, after which the cycle restarts [18].

Besides the functions described above, BAs identify as signaling molecules that bind to a membrane receptor, such as Takeda G-protein receptor 5 (TGR5), and a nuclear hormone receptor, such as farnesoid X receptor-*α* (FXR*α*) [18]. Although BAs bind to several receptors, including sphingosine-1-phosphate receptor 2, muscarinic receptors M2 and M3, formyl peptide receptor 1, liver X receptors *α* and *β*, VDR, pregnane X receptor, and constitutive androstane receptor, TGR5 and FXR*α* are specific receptors that are expressed at high levels in liver cells [8, 42]. When BAs activate TGR5 and FXR*α*, cascade signals introduce the physical stimulations into immune cells and hepatocytes that affect the metabolic routes, including enzymes and transporters of BA metabolism, lipid and glucose metabolism, and inflammation and cancers [8, 18].

BAs are closely associated with HCC [43]. They engage in the carcinogenesis of HCC by directly binding to the receptors and activating signaling pathways that induce changes in the local immune microenvironment and metabolic status of liver cells and cause DNA damage [43].

FXR gene deficiency increases the proinflammatory cytokine IL-1*β* level and elevates the oncogene c-Myc level [32]. FXR is distributed in hepatocytes; FXR agonists are CA, CDCA, LCA, and DCA [42]. TGR5 is expressed on the cell surfaces of the ileum, gallbladder, adipose tissues, and macrophages; TGR5 agonists are LCA and DCA [42]. Evidence reports that TGR5 is an inflammatory suppressor [34]. Activation of TGR5 suppresses LPS-induced production of proinflammatory cytokines and antagonizes NF-*κ*B signaling via the prevention of phosphorylation of I*κ*B*α* (an inhibitor of NF-*κ*B translocation), an important inflammatory pathway [34]. In addition, TGR5 gene deficiency elevates cytokine and chemokine levels, including IL-1*β*, TNF*α*, IL-6, IFN, and MCP-1 [34]. Furthermore, FXR negatively regulates the NF-*κ*B pathway, which has a close relationship with chronic liver inflammation [34]. TGR5 and FXR play vital roles in protecting the liver from inflammation, chronic injury, and cancer.

However, cholesterol and BAs are toxic to tissues and cells. Hydrophobic and hydrophilic BAs have different roles in stimulating cells. A recent study reported that cholesterol accumulation in hepatocytes increased local inflammation and fibrosis through stabilizing TAZ, a transcription factor controlling the expression of genes associated with inflammation and fibrosis [44]. CYP7A1 drives BA metabolism, reducing the deposition of cholesterol in the liver.

DCA and CDCA induce oxidative DNA damage, resulting in their involvement in tumor initiation, and antioxidants reduce the carcinogenic effects [45]. In addition, DCA increases nitrosative stress, resulting in damage to the cellular membrane and DNA [46]. The changes in the constitution of BAs are associated with liver fibrosis. For example, decreased CA and increased CDCA are associated with nonalcoholic steatohepatitis, which may result in altered gut microbiota in patients [47]. The interaction between BAs and gut microorganisms is complicated to determine which one is first. However, the altered composition of BAs or gut microbiota can affect the liver dramatically.

## 5. Conclusion

In the present study, two aspects of an apparent phenomenon were observed. First, upregulated genes that facilitated the transport of BAs were associated with a poor prognosis of HCC in patients. Second, de novo synthesis of BAs benefitted patients with HCC. The reasons may include the following: (1) reabsorbed BAs may hold HCC carcinogens, promoting HCC carcinogenesis; (2) transporters facilitate the accumulation of BAs in hepatocytes, inducing carcinoma development [48]; and (3) recycled BAs feedback to the synthesis of BAs, possibly disrupting the balance of cholesterol and BA metabolism and promoting the aberrant proliferation of liver cells [49]. Concurrently, dysregulation of BA metabolism could activate inflammatory signaling in the liver and increase the risk of HCC development [50]. BA recycling carries many metabolites of gut bacteria into the liver that result in changes in the microenvironment of the liver, leading to carcinogenesis [51]. However, further studies will emphasize the importance of the enterohepatic cycle in liver diseases, including carcinoma.

## Figures and Tables

**Figure 1:** Bile acid-related genes with differential expressions in tumor and nontumor samples. Twenty-six genes were identified with differential expressions (fold change > ∣2∣) (a). Among them, 19 genes were upregulated in tumor samples and 7 genes were upregulated in nontumor samples (*P* < 0.05) (b, c).

**Figure 2:** Annotation and enrichment of 26 identified genes. GO analysis showed that the genes were involved in metabolisms of sterol, monocarboxylic acid, fatty acid, cholesterol, and bile acid and in transports of lipid, organic anion, and bile acid (a). KEGG analysis showed that most of the genes contributed to the ABC transporter family and were involved in the PPAR signaling pathway and syntheses of bile acid, cholesterol, and fatty acids (b).

**Figure 3:** Identification of survival-related genes associated with bile acid metabolism. Twelve genes showed associations with the prognosis of HCC in patients. Among these genes, SLC27A5, CYP7A1, AKR1D1, and ALDH8A1 showed benefits in patients, whereas EFHC1, ABCC1, NPC1, ABCD1, SLC35B2, ABCA4, ABCA3, and SLC51B showed an increased risk of poor prognosis in patients.

**Figure 4:** Three genes for the construction of a prediction model for the prognosis of HCC in patients The expressions of NPC1, ABCC1, and SLC51B in tumor and nontumor samples (a). The distribution of patients with HCC with different risk scores (b). The status of patients with HCC with increasing risk scores (c). The survival curve of the two groups of patients with HCC with high and low risk scores (d).

**Figure 5:** Risk scores and clinical characteristics for the prognosis of HCC in patients. Univariate and multivariate Cox regression analyses of the risk score, age, gender, grade, stage, and T (TNM) for the prognosis of HCC in patients (*P* < 0.001, hazard ratio = 1.568, and 95% CI: 1.256–1.956) (a, b). ROC curve of the risk score, age, gender, grade, stage, and T (TNM) showed that the risk score was more reliable for the prediction of the survival of patients with HCC (AUC = 0.710) (c).

**Figure 6:** Correlation between model genes and clinical characteristics. NPC1 showed differential expression levels in (a) different stages (stage III–IV was higher, *P* < 0.001), (b) grades (grade 3–4 was higher, *P* < 0.001), and (c) TNM (T3–4 was higher, *P* < 0.001). ABCC1 showed higher expressions in high (d) grades, (e) stages, and (f) T (*P* = 0.014, *P* = 0.008, and *P* = 0.016, respectively). Patients with higher risk scores had advanced pathological staging, including the (g) stage, (h) grade, and (i) T (*P* = 0.026, *P* < 0.001, and *P* = 0.027, respectively).

**Table 1:** Three genes identified for the construction of the prediction model.

Genes	Co-ef	HR	HR.95L	HR.95H	*P* value
ABCC1	0.262516	1.300197	1.053752	1.60428	0.014355
NPC1	0.39572	1.485454	1.074874	2.052867	0.016512
SLC51B	0.15545	1.168183	1.046335	1.304221	0.005677

## Data Availability

The datasets used to support the findings of this study are available from TCGA (https://portal.gdc.cancer.gov/repository) database.

## Supplementary Materials

Supplementary Materials Table S1: a total of 127 genes related to the metabolism and transport of bile acid. Table S2: all patients with HCC with risk scores. Fig. S1: GO annotation of the identified genes. The annotation showed that the differential gene expressions were involved in the biological processes, including lipid transport, lipid localization, carboxylic acid synthesis, and fatty acid metabolism; the cellular component, including the basolateral plasma membrane and peroxisomal membrane; and the molecular function, including lipid transporter activity, anion transmembrane transporter activity, and ATPase activity. Fig. S2: analysis of differential gene expressions with GO and KEGG. GO analysis showed that most upregulated genes were involved in ABC transporters and most downregulated genes were involved in primary bile acid biosynthesis (A). KEGG analysis also showed that the genes were involved in the processes of ABC transporters and primary bile acid synthesis (B). Fig. S3: NPC1, ABCC1, and SLC51B showed higher expressions in HCC tissue. NPC1 was stained with HCC (A) and non-HCC tissues (B); ABCC1 was stained with HCC (C) and non-HCC tissues (D); SLC51B was stained with HCC (E) and non-HCC tissues (F). 200x.
